# Intermittent Hydrostatic Pressure Promotes Cartilage Repair in an Inflammatory Environment through Hippo-YAP Signaling *In Vitro* and *In Vivo*

**DOI:** 10.1155/2022/3215461

**Published:** 2022-08-04

**Authors:** Wangxiang Yao, An Ma, Zhen Zhang, Liulong Zhu

**Affiliations:** ^1^Department of Orthopedic Surgery, Affiliated Hangzhou First People's Hospital, Zhejiang University School of Medicine, Zhejiang, China; ^2^School of Basic Medical Sciences & Forensic Medicine, Hangzhou Medical College, Zhejiang, China; ^3^Department of Orthopedic Surgery, Hangzhou Orthopedic Institute, Affiliated Hangzhou First People's Hospital, Zhejiang University School of Medicine, Hangzhou, China

## Abstract

The study of chondrogenic progenitor cells (CPCs) as seed cells has become a new focus of cartilage regeneration. The inflammatory environment of osteoarthritis (OA) inhibits the repair ability of CPCs. But the OA patients' CPCs showed an excellent regeneration ability with intermittent hydrostatic pressure (IHP). However, the mechanism is unclear. We compared the expression of the Hippo signaling effect factor YAP between OA and normal cartilages. Then, the relationship between the Kellgren-Lawrence (K-L) score of OA and the rate of YAP-positive cells was analyzed. The changes of CPCs after IHP and IL-1*β* applications were observed. The OA model was established by cutting the anterior cruciate ligament of rats. The knee joint of the OA rats was distracted by hinged external fixator to create suitable IHP, named as the IHP group. The IHP group plus intra-articular injection of Verteporfin (VP) was named as the IHP+VP group, and the untreated rat group was named as the CON group. Four and 8 weeks after the operation, the reparative effect was evaluated by MASSON staining and immunohistochemical staining. Lower levels of YAP1 and higher expressions of p-YAP1 were found in the OA group as compared to the normal group. IHP inhibited the Hippo signaling in an inflammatory environment and promoted the proliferation of CPCs. The cartilage deterioration in the CON group progressed more significantly than that in the IHP+VP group. The best reparative effect was observed in the IHP group with increased expression of YAP1 and decreased p-YAP1. These results hint that mechanical stress can activate CPCs and promote cartilage repair in an inflammatory environment through inhibiting Hippo signaling.

## 1. Introduction

As an inflammatory factor in osteoarthritis (OA), IL-1*β* plays a major role in OA cartilage destruction, which inhibits the proliferation of chondrocytes, induces apoptosis, causes the degradation of cartilage extracellular matrix, and aggravates cartilage erosion [1]. Recently, chondrogenic progenitor cells (CPCs) as adult stem cells have been paid more attention for their long lasting chondrogenic differentiation potential under suitable conditions [2, 3]. However, under the inflammatory environment of OA with the presence of IL-1*β*, the ability of CPCs to migrate from deep zone to surface to repair cartilage was inhibited, leading to the failure of cartilage regeneration [4]. Cartilage was mainly regulated by mechanical stress because loading was essential to maintain tissue adaptation and remodeling [5]. Our previous studies showed that intermittent hydrostatic pressure (IHP) can promote the migration of CPCs and increase their proliferation ability [6], but it is unclear whether the same effect can be achieved in an OA inflammatory microenvironment.

Yes⁃associated protein (YAP) is an effector protein downstream of Hippo signaling and a transcriptional cofactor considered as one of major cellular mediators which define the cell fate [7]. YAP signaling may represent a vital mediator that maintains the constant adaptation of bone and cartilage tissues in response to changes of the mechanical environment [8, 9]. For example, homogenous shear stress can inhibit an inflammatory response through YAP and thereby act as major protagonists in the maintenance of tissue homeostasis [10]. Also, abnormally increased mechanical stress in the joint of OA patients may activate the Hippo signaling, then NF-*κ*B signaling to regulate the expression of proteases and the cartilage degradation. In addition, inflammatory cytokines such as IL-1*β* can trigger YAP degradation through TAK1-mediated phosphorylation during osteoarthritis, thus linking the inflammation to the mechanical stress [11]. However, it is unclear whether YAP could be activated in the CPCs under the action of IHP to regenerate cartilage in an inflammatory environment.

For joint distraction, the two bony ends of a joint are gently separated and held apart for a certain distance through an external fixation frame [12]. Loading during the joint distraction leads to the pressure oscillations of the joint fluid when two ends of the bone approach towards each other, which is used for treating posttraumatic arthritis and to explore the mechanism of IHP *in vivo* [13]. The joint distraction reduced the secondary inflammation level, cartilage degeneration, and subchondral bone sclerosis followed with a slow OA progression [14]. Also, increased synthesis of collagen type II and hyaline cartilage nature of the newly regenerated tissue by the joint distraction were observed through an arthroscopic observation [15]. However, the mechanism of joint distraction that leads to tissue repair is still unclear.

In this paper, we compared the cartilage YAP expression levels between normal and OA patients and examined its correlation with the severity of OA by immunohistochemical staining and western blot analysis firstly. Secondly, the CPCs from the OA patients were extracted, cultured, and amplified and then cultured on the scaffold constructed by alginic acid. We then observed the changes of Hippo signaling under IHP in the inflammatory environment created by IL-1*β*. Thirdly, the OA model was established by cutting the anterior cruciate ligament (ACL) of rats, and IHP was created by means of knee joint distraction with hinged external fixator to observe the reparative mechanism. Therefore, the first purpose of this study was to determine whether YAP could modulate the cartilage metabolism in the osteoarthritic joint and contribute to the disease progression. Then, the secondary objective was to explore the mechanism on how IHP promotes the repair of OA cartilage in vitro and in vivo through Hippo signaling.

## 2. Materials and Methods

### 2.1. Harvesting and X-Ray Evaluation of Osteoarthritic Cartilage

The cartilage used in this project was collected from the OA patients with knee posttraumatic arthritis at the same hospital from September 2014 to December 2019. This project had received the consent from the patients and the approval of the hospital ethics committee (Hangzhou First People's Hospital, No. 309). There were 26 OA patients (mean age of 56.4 ± 12.1 years) named as the OA group. The Kellgren-Lawrence (K-L) score of knee-standing X-ray was used to evaluate the severity of OA. Twelve patients without joint degeneration (mean age 57.4 ± 10.9 years) were enrolled as the control group and operated on for the femoral neck fracture.

### 2.2. CPC Procurement and 3D *In Vitro* Cell Culture Model Preparation

CPCs were isolated from the OA patients and cultured as described before [16]. In brief, under sterile conditions, trypsin digestion and mechanical dissociation were adopted to isolate cells from the cartilage. After counting and centrifuging, the CPCs were resuspended in fresh DMEM/F12 with 10% FBS (Sigma-Aldrich, Milan, Italy). The medium was changed after 24 h and twice per week thereafter. These CPCs were passaged routinely when they reached 70% confluence. The passage 2 (P2) was used for 3D culture.

A 3D in vitro cell culture model was performed as reported by us before [6]. Briefly, the CPCs were suspended in 2% (*w*/*v*%) alginate solution (Sigma-Aldrich, Milan, Italy) at a density of 8 × 10^5^ cells/ml, then added into the CaCl_2_ solution (100 mmol/l) dropwise. The cell-laden alginate beads were then incubated in fresh DMEM/F12 with 10% FBS for 7 days before the successive experiments. As described before [17], we used 0.01 ng/ml IL-1*β* (Sigma-Aldrich, Milan, Italy) to mimic the inflammatory environment.

### 2.3. *In Vitro* IHP Model Preparation

The IHP model was established by us before [6]. A special device which generates IHP with a defined frequency (0.1–1 Hz) and amplitude (0.2–10 MPa) was produced by the Taixing Experimental Instrument Factory (Taixing, Nanjing, China). The amplitude and frequency were set at 5 MPa and 0.5 Hz for 4 h/day [18]. All experiments were performed on three sets of samples for statistical validation.

Based on the published articles, we chose Verteporfin (VP) to inhibit the Hippo signaling pathway by interrupt TEAD–YAP interaction [19]. When VP (Selleck, shanghai, China) was added to the medium, the cell proliferation was significantly suppressed, and the inhibitory effect was different at different concentrations. Finally, 20 *μ*M was selected as the working concentration. VP was dissolved in DMSO and added to the DMEM/F12 with 10% FBS for the proliferation assay immediately or incubated with the CPCs for 30 min prior to the subsequent western blot experiment.

### 2.4. Western Blot Analysis

Tissue samples were collected and lysed with M-PER mammalian protein extraction reagent buffer (Thermo Fisher Scientific, San Jose, CA, USA) containing protease inhibitor cocktail (Thermo Fisher Scientific, Rockford, Illinois, USA) in ice-cold temperature. After 30 min of lysis, the proteins were extracted by centrifugation at 13,000 g for 15 min. The protein concentrations were determined using the BCA protein assay kit (Thermo Fisher Scientific, San Jose, CA, USA). Equal amounts of protein (40 *μ*g) from each sample were separated with 10% sodium dodecyl sulphate–polyacrylamide gel electrophoresis (SDS–PAGE) and electrophoretically transferred to PVDF membranes (Millipore, Boston, MA, USA) for immunoblotting. After being blocked with 5% nonfat milk in TBST for 1 h at room temperature, the blots were incubated overnight at 4°C with primary antibodies against human YAP1 (1 : 1000, ET1608-30), p-YAP1 (1 : 1000, ET1611-69), and GAPDH (1 : 5000, EM1101). All antibodies were obtained from Huabio Technology (Hangzhou, China). The immunoreactive protein blots were visualized using SuperSignal reagents (ECL; Millipore, Billerica, MA, USA), and the results were analyzed with ImageJ software.

### 2.5. Flow Cytometry Assay

The P2 CPCs were retrieved from the 3D in vitro chondrocyte culture model by adding 55 mM Na citrate at a volume of 4-5 times that of the beads. The cells were spined down by shaking for 20-30 min. After fixed with 70% ethanol, the cells were stained and treated with propidium iodide for cell cycle analysis. Flow cytometry as a cell cycle assay was performed on FACSVerse (BD Biosciences) according to the manufacturer's instructions, and the results were analyzed using FlowJo software (version 7.6.2; Tree Star).

### 2.6. Electron Microscope and Immunofluorescence Assay Analysis

The cell alginate microspheres were washed with PBS for 3 times, then added to 2.5% glutaraldehyde solution and fixed at 4°C, dehydrated, embedded, stained with lead citrate solution and uranic acetate dioxide, and sliced into ultrathin slices with Leica EMUC7. At least 100 CPCs from each group were evaluated, and a single cell containing more than 5 vacuoles in the cytoplasm was defined as the vacuolated cell [20].

For the immunofluorescence assay, the anti-YAP1 antibody was used as the preliminary with a dilution of 1 : 25, and the goat polyclonal secondary antibody to rabbit IgG-H&L (Alexa Fluor® 488) was used as the secondary antibody. The positively stained cells were counted in a field of 50 × 50 *μ*m grid (40x field), and the positive staining rate was determined as the number of positively stained cells in 5 fields/total number of cells in the field of view × 100%.

### 2.7. RT-qPCR

Total cellular RNA was extracted using TRIzol (Invitrogen, California, USA). Using PrimeScript RT reagent kit (Takara, Tokyo, Japan), 1 *μ*g total RNA was used to make cDNA. The SYBR Green Real-Time PCR Master Mix kit (Takara, Tokyo, Japan) was used to perform the RT-qPCR reactions on ABI-7500 Real-Time PCR Systems (Applied Biosystems, Massachusetts, USA). The qPCR primers of different genes are listed in Table 1.

The relative gene expression level was calculated by the normalization to the expression level of GAPDH using the 2-*ΔΔ*ct method. All experiments were performed in triplicate and analyzed with the GraphPad Prism program.

### 2.8. In Vivo IHP Model Preparation

All animal experiments were approved by the animal ethics committee of Zhejiang Chinese Medical University. The 8-week-old (200–250 g, male) Sprague-Dawley rats were provided by the Animal Experiment Center of Zhejiang Chinese Medical University. The in vivo IHP model was made by us with some minor modifications according to the method reported by Chen et al. [14]. The ACL of the rats was transected for 4 weeks, the posttraumatic OA was successfully induced, and the distraction arthroplasty was performed by hinged external fixators (Xinzhong Biological Instrument, Tianjing, China). Briefly, a total of three pins (1.2 mm in diameter) was manually drilled into the lateral side of the knee joint, one in the lateral femoral epicondyle, the other two in the proximal tibia. Finally, the joint space was widened for 1 mm by the external fixator. All animals were allowed to move freely during the successive eight weeks of the study.

All posttraumatic OA rats were divided into 3 groups randomly: one control group without IHP treatment (CON group), one IHP treatment group (IHP group), and one group treated with IHP combined with VP (IHP+VP group) (*n* = 10). Alginate beads soaked with VP (5 *μ*g/rat) were implanted into the knee joint cavity of the OA mice immediately after IHP treatment [11]. All animals were euthanized 4 or 8 weeks later.

### 2.9. ELISA Assay of IL-1*β*

Eight weeks after the joint distraction, the rats were euthanized, and one milliliter of serum was collected by cardiac puncture with a sterile syringe. All serum samples were centrifuged at 1000 × g for 10 min and stored at −80°C until ELISA assay. The rat IL-1*β* high-sensitivity ELISA kit (70-EK301BHS-96, Multisciences Biotech, China) was used to quantify the IL-1*β* level with a microplate reader (MK3, Thermo, USA). All experiments were repeated three times.

### 2.10. Histological and Immunohistochemical Assay

Clinically, we harvested the cartilage samples from the degenerated area on the femoral condyles using a custom-made biopsy device. The animal cartilage samples were harvested from the femoral condyles of knees and fixed with 4% paraformaldehyde, then sliced into paraffin sections according to the standard protocol. The MASSON staining was used for the histological examination, and the Mankin scores were used to evaluate the regenerated cartilage in vivo by two independent blinded observers. For the immunohistochemical assay, rabbit antirat YAP1, p-YAP1, and MMP13 antibodies (Huabio Technology, Hangzhou, China) were used with a dilution of 1 : 50 overnight at 4°C, and the enzyme-labeled goat antirabbit IgG polymer (Huabio Technology, Hangzhou, China) was used as the secondary antibody. Finally, the sections were counterstained with hematoxylin. The rates of the positively stained cells were calculated as described above.

### 2.11. Statistical Analysis

All statistical analyses were performed using the statistical software SPSS13.0. The data were analyzed via one-way ANOVA followed by Turkey's test. The assumptions of the analysis were assessed by the Shapiro-Wilk test of normality and Levene's test for homogeneity of variance. The result of Levene's test was used to determine the post hoc testing strategy. The values of *P* < 0.05 in the statistical comparisions were considered as significantly different. Data were reported as mean and 95% CI (confidence interval).

## 3. Results

### 3.1. Abnormal Expressions of YAP and p-YAP in OA Patients and Their Association with the K-L Score

The expressions of YAP and p-YAP were explored by western blot and immunohistochemical staining analysis (Figures 1(b)–1(f)). Lower expression levels of YAP and higher expression levels of p-YAP were found in the OA group as compared to the control group (Figures 1(b)–1(e)) (*P* < 0.0001, respectively). Additionally, these expressions had a good correlation with X-ray evaluation (K-L scores) (Figure 1(a)) since the lower YAP expression and higher p-YAP expression found in the OA group had higher K-L scores (Figures 1(c), 1(e), and 1(f)) (*P* < 0.0001, respectively).

### 3.2. Mechanical Stress Inhibits the Hippo Signaling in an Inflammatory Environment and Promotes the Proliferation of CPCs

The flow cytometry assay showed that the percentage of CPCs in the G2+S phase increased with IHP, while the percentage of CPCs in this phase decreased after applying VP (Figure 2(a)). HE staining found the morphology of the CPCs changed after adding IL-1*β*, showing shrinkage (Figure 2(b)). Also, under an electron microscope, the mitotic phase was reduced, the endoplasmic reticulum was not obvious, and apoptotic bodies and many vacuoles were formed after adding IL-1*β*. However, after applying IHP, the cell morphology became normal and the vacuoles were reduced, the mitotic phase increased, and the endoplasmic reticulum clearly proliferated. While applying VP in the IHP group, the cells were improved, some vacuoles were formed, and endoplasmic reticulum hyperplasia was observed (Figures 2(c) and 2(d)) (*P* < 0.05, respectively).

After adding IL-1*β*, the expression of YAP in CPCs decreased, and only a small amount of YAP was expressed in the nucleus (the positive rate of nucleus was 25%). After applying IHP, the expression of YAP increased, in particular in the nucleus (the positive rate of nucleus was 46%) (Figures 2(e) and 2(f)) (*P* < 0.001). This suggests that the transfer of YAP from the cytoplasm to the nucleus could initiate downstream gene expression and promote CPC proliferation. The western blot analysis showed that the IL-1*β* treatment decreased the YAP expression and increased the p-YAP expression (Figure 2(g)). Interestingly, IHP did not alter the expression of YAP at 30 min but increased the YAP expression at 60, 120, and 240 min, which indicates that the mechanical stress needed a certain time to influence YAP and p-YAP expression. Furthermore, IHP increased the proliferation and cartilage differentiation of genes, such as Sox-9, Aggrecan, Col 2A, CTGF, cyclin, and YAP, and decreased the expression of Col 1A and Runx-2, while adding VP decreased the expression of Sox-9, Aggrecan, Col 2A, CTGF, cyclin and YAP, and increased the expression of Runx-2 (Figure 2(h)).

### 3.3. Joint Distraction Promotes OA Cartilage Repair In Vivo

The rats were killed four weeks after ACL transection. The cartilage on the load-bearing surface of the femoral medial condyle and tibial plateau was slightly eroded and worn, showing typical OA-like changes as described by us before [16]. The serum IL-1*β* concentration was increased in the CON group and reduced in the IHP group (Figure 3(a)).

In the IHP group, the cartilage surface fibrosis decreased after 4 weeks of the distraction, but there were still defects and cracks, and the chondrocytes arranged orderly. After 8 weeks, the cartilage surface fibrosis decreased further, and the chondrocytes arranged in order and secreted more extracellular matrix, which basically repaired the cartilage. In the CON group, cartilage repair was rare after 4 weeks and many fibrous tissues proliferated; also, the layers of cartilage lost their normal arrangement. Then, after 8 weeks, the proliferation of fibrous cartilage decreased, but the cells were still disordered and displayed typical OA changes. In the IHP+VP group, the cartilage surface degenerated, the cells were disordered, and the trabeculae were sparse after 4 weeks. By 8 weeks, some fibrocartilage tissues were formed, chondrocytes were disordered, and a small amount of extracellular matrix was secreted. The Mankin scores at different time points showed significant differences among the treatment groups. The IHP group scored the lowest, while the IHP+VP group scored lower than the CON group (Figure 3(b)) (*P* < 0.05, *P* < 0.01, respectively).

### 3.4. Joint Distraction Decreased p-YAP and Increased YAP Expression

In the CON group, only a small amount of YAP expression was found in the deep zone and not significantly different between 4 and 8 weeks. In the IHP+VP group, a small amount of YAP expression was observed after 4 weeks and slightly increased after 8 weeks. In the IHP group, more YAP was expressed in the nucleus of cartilage cells after 4 weeks and was mainly distributed either on the surface or around the proliferating cells, and the YAP expression increased further after 8 weeks (Figure 3(c)). Statistical analysis of the rates of the YAP-positive cells showed that the IHP group had the significantly highest positive rate (*P* < 0.05 and *P* < 0.01, respectively).

In the CON group, the expression of p-YAP increased clearly in the deep zone and was mainly expressed in cytoplasm after 4 weeks as well as after 8 weeks. In the IHP+VP group, the expression of p-YAP was mainly in the superficial zone after 4 weeks but less than that in the CON group and decreased after 8 weeks. In the IHP group, partial expression of p-YAP was found in the superficial zone after 4 weeks but decreased after 8 weeks (Figure 3(d)). Statistical analysis of the rates of the p-YAP stained cells showed that the rate in the CON group was the highest, followed by that in the IHP+VP group, while the IHP group had the lowest rate, with statistical significance between groups (*P* ≤ 0.001 and *P* < 0.0001, respectively).

### 3.5. Joint Distraction Decreased the Expression of MMP13

MMP13 was mainly expressed in the degenerated extracellular matrix of the CON group and increased further after 8 weeks. In the IHP group, a small amount of MMP13 expression was found in the subchondral bone and medullary cavity after 4 weeks but was not obvious in the superficial zone, and the MMP13 expression was further reduced after 8 weeks compared with that in the CON group. The MMP13 expression in the IHP+VP group was less, distributed in the deep zone, and decreased after 8 weeks, mainly in the medullary cavity (Figure 3(e)). Statistical analysis of MMP13-expressed cells showed that the positive rate in the CON group was the highest, followed by that in the IHP+VP group, and the lowest in the IHP group, with statistical significance (*P* ≤ 0.01 and *P* < 0.001, respectively).

## 4. Discussion

The recently discovered CPCs from cartilage of OA patients provided new possibilities for the treatment of OA [21]. Our previous experiments confirmed that the chondrogenic ability of the CPCs cultured in vitro is better than that of synovial stem cells and chondrocytes [6]. Therefore, we continued to use the CPCs to explore its chondrogenic ability under an inflammatory environment in order to provide theoretical basis for its clinical application in the treatment of OA. Although the CPCs metabolism was affected by various physical, chemical, and biological factors, mechanical factors may play a more important role [22]. For example, low-frequency and high-intensity mechanical stress can induce OA progression by activating p38-MAPK and cause upregulation of inflammatory factors [23]. In this experiment, the intermittent hydrostatic pressure of 5 MPa and 0.5 Hz lasting for 4 hours and the 3D culture mode using alginic acid as scaffold were used to simulate the environment of CPCs in vivo, which provides a suitable model for further study [24].

Previous studies have shown that the Hippo pathway keeps cartilage hemostasis by controlling chondrocyte differentiation and endochondral ossification, thus playing an important role in cartilage metabolism after birth [25]. The expression of YAP in the mouse knee joints gradually decreased with age [11]. Interestingly, after balancing the age factors, we found that the expression of p-YAP increased and YAP decreased in the OA group compared to those in the control, indicating that the activation of the Hippo pathway is related to the progression of OA. With increased K-L scores, the expression of YAP also decreased, suggesting that the activation degree of the Hippo pathway is positively correlated with the severity of OA.

OA is mainly expressed as the destruction of chondrocytes and the extracellular matrix, leading to dysfunction, in which inflammatory factors play a major role [26]. IL-1*β* is considered as an important inflammatory factor in the pathogenesis of OA and is widely used to construct an inflammatory environment [27, 28]. When IL-1*β* was added to the culture medium, the proliferation ability of CPCs was weakened, and the expression of YAP was reduced. Under an electron microscope, the vacuoles in the cytoplasm were clearly increased, indicating an endoplasmic reticulum stress or autophagy, which suggests that the cells were in an inhibitory state [20]. Also, when using VP to inhibit YAP's effect, OA articular cartilage was continuously degraded [11]. However, the activation of YAP gradually increased after applying IHP, which could resist IL-1*β*-mediated inhibitory conditions and promote CPC proliferation. When VP was used to block the combination of YAP and its effector, the cells were partially in the inhibited state again, which proved that YAP promotes the CPC proliferation. The increased expression of YAP in CPCs and the increasing entry of YAP into nucleus after compression as shown by the immunofluorescence staining intuitively demonstrated the shuttle mechanism of YAP under mechanical stress. Our results showed that mechanical stress promoted the CPC proliferation through regulating the activity of YAP, and the YAP entering the nucleus could activate the expression of the downstream genes to promote the CPC proliferation [29]. It was previously showed that mechanical stress activated the expression of YAP to promote the repair of lung injury in a mouse pneumonectomy model [30]; thus, YAP may play a decisive role in cell fate determination under OA inflammatory environments.

Although recent studies have confirmed the promotion of the chondrogenic differentiation of CPCs by mechanical stress [5, 8, 24], the mechanism has not been reported. Low expression of Sox-9 in CPCs of OA patients leads to a decline of their ability to repair cartilage [2]. CTGF is an important downstream gene of YAP, which can promote the proliferation of stem cells to repair tissues [31]. In this experiment, it was observed that the expression of Sox-9 and CTGF increased after being pressurized with IL-1*β* but decreased after VP was applied. It was reported that Sox-9 and Runx-2 regulated the differentiation direction of CPCs, and the knocking out of Runx-2 promoted the cartilage differentiation ability [2]. We also observed the decreased expression of Runx-2 by IHP, and its expression increased after VP was applied. It was reported that YAP could promote endochondral ossification and affect fracture healing by combining with Runx-2 [25]. Our results indicate that appropriate IHP could promote the cartilage differentiation and the chondrocyte proliferation by upregulating Sox-9 and CTGF and downregulating Runx-2 in an inflammatory environment created by IL-1*β* in vitro.

To further verify the effect of IHP on cartilage metabolism in vivo, we provided a suitable IHP through joint distraction with an external fixator [15]. Because CPCs are MSC-like stem cells, the existence of CPCs in the articular cartilage was considered as the main reparative cells to maintain the metabolism of the joint through local proliferation or apoptosis [2, 32]. We found increased expression of p-YAP and the inhibited condition of cells in the control group, indicating that CPCs repairing ability was also decreased, leading to a deterioration in cartilage repair. A study confirmed that the proliferation of synovial stem cells was YAP-dependent [33]. Hence, the results of the cartilage repair in the joint distraction group accompanied by increased expression of YAP and decreased expression of p-YAP indicate that IHP can inhibit Hippo signaling in vivo to promote cartilage repair. The process of repairing cartilage may be completed by CPCs proliferation and differentiation to chondrocytes [2]. However, due to the limitation of observation methods, we have not observed the change of YAP expression in CPCs after joint distraction, and further experiments are needed to verify it.

MMP13 is one of the main degradation enzymes that cause OA cartilage destruction [34]. It is mainly expressed in the superficial and deep layers of OA cartilage and is often related to the disordered extracellular matrix. The reduced expression of MMP13 in the IHP group revealed that an appropriate mechanical stress could protect cartilage by inhibiting the expression of degradation enzymes. Also, the decreased serum IL-1*β* concentration in the IHP group may be caused by the improved condition of OA.

To sum up, Hippo signaling plays an important role in maintaining cell homeostasis of articular cartilage, and mechanical stress can promote cartilage repair in an inflammatory environment by activating CPCs to express YAP, which provides a new target for the treatment of OA.

## Figures and Tables

**Figure 1:** (a) The knee standing X-ray images of OA patients at different stages (the Kellgren-Lawrence score I-IV). (b) Immunohistochemistry staining images of YAP expression in the articular cartilage cells between the OA and control groups. (c) The significantly positive correlation of YAP^+^ chondrocytes in the OA group with the K-L score negatively (*P* < 0.0001). (d) Immunohistochemistry staining images of p-YAP expression in the articular cartilage cells between the OA and control groups. (e) The significantly positive correlation of p-YAP^+^ chondrocytes in the OA group with the K-L score (*P* < 0.0001). (f) Western blotting images of YAP1 and p-YAP1 expressions of the OA and control groups. (g) Western blotting images of YAP1 in the OA group and the negative correlation with the K-L scores (*P* < 0.0001).

**Figure 2:** (a) Flow cytometry to detect cell cycle after IHP and IL-1*β* applications. (b) H&E staining of CPCs after IHP and IL-1*β* applications (bars: 40 *μ*m). (c) Electron microscopic image of CPCs after IHP and IL-1*β* applications. (d) Vacuolated cell rate of CPCs after IHP and IL-1*β* applications (*n* = 4, ^∗^*P* < 0.05). (e) YAP immunohistochemical assay images of CPCs after IHP and IL-1*β* applications. (f) Analysis of YAP-positive CPCs after IHP and IL-1*β* applications (*n* = 4, ^∗∗∗^*P* < 0.001). (g) Western blot images of CPCs after IHP and IL-1*β* applications. (h) RT-qPCR gene expression of CPCs after IHP and IL-1*β* applications.

**Figure 3:** (a) The serum IL-1*β* concentration in each group after eight weeks of the operation. (b–e) MASSON, YAP1, p-YAP1, and MMP13 immunohistochemical staining of regenerated cartilage in each group at each time point after the operation. The results are presented as the mean ± SD (*n* = 4, ^∗^*P* < 0.05, ^∗∗^*P* < 0.01).

**Table 1:** The qPCR primers of different genes.

Gene	5′ to 3′ sequence	
*Col1A1*	Forward	GAGGGCCAAGACGAAGACATC
	Reverse	CAGATCACGTCATCGCACAAC

*Col2A1*	Forward	TGGACGCCATGAAGGTTTTCT
	Reverse	TGGGAGCCAGATTGTCATCTC

*Aggrecan*	Forward	CCCCTGCTATTTCATCGACCC
	Reverse	GACACACGGCTCCACTTGAT

*Sox-9*	Forward	AGCGAACGCACATCAAGAC
	Reverse	CTGTAGGCGATCTGTTGGGG

*Runx-2*	Forward	GGACCTCGGGAACCCAGAAG
	Reverse	ACTTGGTGCAGAGTTCAGGGA

*CTGF*	Forward	ACCGACTGGAAGACACGTTTG
	Reverse	CCAGGTCAGCTTCGCAAGG

*YAP1*	Forward	TAGCCCTGCGTAGCCAGTTA
	Reverse	TCATGCTTAGTCCACTGTCTGT

*Cyclin*	Forward	CTGCGCGAGAAGGAACTGAA
	Reverse	GTCTACAAAGAATCGACGGCTC

*GAPDH*	Forward	AGGTCGGTGTGAACGGATTTG
	Reverse	GGGGTCGTTGATGGCAACA

## Data Availability

All data generated or analyzed during this study are included in this published article.

## Abbreviations

OA: Osteoarthritis
IHP: Intermittent hydrostatic pressure
YAP: Yes-associated protein
ACL: Anterior cruciate ligament.
